# Sulforaphane Upregulates Cultured Mouse Astrocytic Aquaporin-4 Expression through p38 MAPK Pathway

**DOI:** 10.1155/2022/1144124

**Published:** 2022-08-10

**Authors:** Canhong Yang, Sisi Qin, Jiafa Zhang, Yuanyuan Wang, Huan Li, Tianming Lü

**Affiliations:** ^1^Department of Neurology, The Third Affiliated Hospital of Southern Medical University, Guangzhou 510630, China; ^2^Department of Critical Care Medicine, The Fifth Affiliated Hospital of Sun Yat-Sen University, Zhuhai 519000, China; ^3^Department of Neurology, Nansha Hospital, Guangzhou First Peoples Hospital, School of Medicine, Southern China University of Technology, Guangzhou 510630, China

## Abstract

Protein misfolding and/or aggregation are common pathological features associated with a number of neurodegenerative diseases, including Alzheimer's disease (AD) and Parkinson disease (PD). Abnormal protein aggregation may be caused by misfolding of the protein and/or dysfunction of the protein clearance system. Recent studies have demonstrated that the specific water channel protein, aquaporin-4 (AQP4), plays a role in the pathogenesis of neurodegenerative diseases involving protein clearance system. In this study, we aimed to investigate the role of sulforaphane (SFN) in the upregulation of AQP4 expression, along with its underlying mechanism using cultured mouse astrocytes as a model system. At low concentrations, SFN was found to increase cell proliferation and result in the activation of astrocytes. However, high SFN concentrations were found to suppress cell proliferation of astrocytes. In addition, our study found that a 1 *μ*M concentration of SFN resulted in the upregulation of AQP4 expression and p38 MAPK phosphorylation in cultured mouse astrocytes. Moreover, we demonstrated that the upregulation of AQP4 expression was significantly attenuated when cells were pretreated with SB203580, a p38 MAPK inhibitor. In conclusion, our findings from this study revealed that SFN exerts hormesis effect on cultured mouse astrocytes and can upregulate astrocytic AQP4 expression by targeting the p38 MAPK pathway.

## 1. Introduction

Insoluble protein deposits in the brain formed by soluble peptides or proteins are a common pathological hallmark of neurodegenerative diseases, including Alzheimer's disease (AD), Huntington's disease (HD), and Parkinson disease (PD) [1]. Misfolding and/or aggregation of *β*-amyloid (A*β*) peptide and tau protein is associated with AD [2], while the abnormal aggregation of *α*-synuclein and tau protein is related to PD [3]. Abnormal protein aggregation is typically thought to be caused by misfolding of the protein and/or dysfunction of the protein clearance system. In the case of AD, A*β* clearance is thought to be a central player around which multiple factors involved in the development of disease revolve [4]. Thus, novel targets that function to enhance A*β* clearance may represent promising future strategies for the treatment of AD. Clearance of A*β*, tau, and other proteins in brain parenchyma can occur through several different pathways but primarily involves the blood-brain barrier (BBB) pathway, the enzyme/glial degradation pathway, and the central nervous system (CNS) lymphatic drainage system [5]. To date, according to current studies, the CNS lymphatic drainage system at least consists of the perivascular drainage pathway [6], the glymphatic system [7], and the dural lymphatic vascular system [8, 9]. In glymphatic system, subarachnoid space cerebrospinal fluid (CSF) enters into the brain parenchyma along para-arterial Virchow-Robin spaces (VRS) and mixes with interstitial ﬂuid (ISF), the CSF-ISF, and then returns to the subarachnoid space along paravenous VRS, entering the bloodstream or reaching the cervical lymphatic system through the dural lymphatic vessels around arteries and sinuses. Thus, interstitial ﬂuid and waste solutes can be cleared with ISF bulk ﬂow [7, 10]. Studies have demonstrated that aquaporin-4 (AQP4), a specific water channel protein, plays an important role in the clearance function of glymphatic system [7]. AQP4 has been demonstrated to be the most predominant aquaporin protein found in the mammalian brain. It is primarily distributed on the endfeet of astrocytes, which is associated with astrocytic polarity and function [11]. AQP4 has also been shown to play an important role in the pathophysiological processes of encephaledema, brain tumors, epilepsy, and neuromyelitis optica [12]. Accumulating evidence from a number of studies has demonstrated that AQP4 plays a role in the pathogenesis of neurological degenerative diseases, including AD [5, 13]. This evidence suggests that AQP4 could provide a novel target for the prevention and treatment of these diseases.

Sulforaphane (SFN) is a type of isothiocyanates and is widely prevalent in the brassicaceous vegetable. Interestingly, SFN has been shown to possess potential antitumor [14], antibiosis [15], and antioxidant [16] properties. In addition, SFN has been demonstrated to exert neuroprotective effects in the case of stroke, traumatic brain injury (TBI), and neurodegenerative diseases [17]. Previous research has shown that SFN has the ability to upregulate AQP4 expression in TBI animal models [18]. However, the underlying mechanism by which this occurs remains unknown. In this study, we aim to explore the effect of SFN on the upregulation of astrocytic AQP4 expression in cultured mouse astrocytes, as well as the mechanism surrounding this regulation of AQP4 expression. We demonstrated that SFN functions to upregulate astrocytic AQP4 expression by targeting the p38 MAPK pathway. To the best of our knowledge, this work represents the first study aimed at revealing this underlying mechanism of the effect of SFN on astrocytic AQP4 expression.

## 2. Materials and Methods

### 2.1. Reagents and Antibodies

SFN was purchased from Aladdin (China). The CCK-8 assay kit was purchased from Dojindo (Japan). FITC Annexin V Apoptosis Detection Kit I was purchased from BD Biosciences (USA). DNase I was purchased from Sigma (USA). The TUNEL apoptosis detection kit and DAPI were purchased from Beyotime (China). DMEM/F12 medium, fetal bovine serum (FBS), 25% (w/v) trypsin-EDTA, Phosphate Buffered Saline (PBS), goat serum, Alexa fluor 594 labeled goat anti-chicken secondary antibodies and Alexa fluor 488 labeled goat anti-rabbit secondary antibodies, RIPA lysis buffer, protein phosphatase inhibitors, BCA protein assay kit, and the ECL reagent kit were purchased from Thermo Scientific (USA). Caspase-3 and cleaved Caspase-3 rabbit polyclonal antibodies, SB203580, p38 MAPK, and phospho-p38 MAPK rabbit mAb were purchased from Cell Signaling Technology (USA). GFAP chicken polyclonal antibody, GFAP rabbit polyclonal antibody, and AQP4 rabbit polyclonal antibody were purchased from Abcam (USA). Beta tubulin rabbit polyclonal antibody and horseradish peroxidase-conjugated goat anti-rabbit secondary antibodies were purchased from Proteintech (USA).

SFN was dissolved in dimethyl sulfoxide (DMSO) to a storage concentration of 100 mM. SB203580 was dissolved in dimethyl sulfoxide (DMSO) to a storage concentration of 10 mM. 0.01%(v/v) DMSO was used as vehicle.

### 2.2. Cell Culture

Astrocytes were cultured from neonatal C57BL/6J mouse (postnatal day 1, purchased from Southern Medical University's Experimental Animal Center). Animal experiments were carried out with approval from the Institutional Animal Care and Use Committee of Southern Medical University in accordance with the guidelines of the Institutional Animal Care and Use Committee as outlined by the National Institutes of Health and the Guide for the Care and Use of Laboratory Animals. Meninges were removed from the brains of neonatal mouse and the cerebral cortices were dissected out and collected in DMEM/F12 medium. Brain tissue was homogenized followed by digestion with 25% (w/v) trypsin-EDTA for 5 minutes at 37°C. The trypsin reaction was terminated by supplementation with DMEM/F12 medium containing 10% (v/v) FBS. The homogenate was then resuspended in serum-free DMEM/F12 containing DNase I, followed by filtration with 75 *μ*m mesh sieves. Filtered homogenate was centrifuged at 200 ×g for 5 minutes. Following centrifugation, the supernatant was discarded and the pellet was resuspended in DMEM/F12 medium containing 10% FBS. Cells were cultured at 37°C in a humidified incubator with 5% (v/v) CO_2_ and cell culture medium was changed every 2-3 days. Astrocyte cultures grew to approximately 80–90% confluency, at which point they were subcultured or used for experiments. Cultured cells were identified using immunofluorescence to stain for the specific astrocytic marker, glial fibrillary acidic protein (GFAP). GFAP staining revealed that the astrocytic cultures were of greater than 99% purity, a level suitable for experiments (Figure 1).

### 2.3. CCK-8 Assay

A CCK-8 kit was used to determine cell proliferation. Second passage astrocyte cultures were seeded into a 96-well plate at a density of 0.5 × 10^4^ cells/well. When cultures grew to approximately 80–90% confluency, complete medium was replaced with serum-free DMEM/F12 for 24 hours and cells were treated with different concentrations of SFN for 6, 12, and 24 hours, respectively. Following SFN treatment, 10 *μ*l of CCK-8 reagent was added to each well, and cells were incubated at 37°C with 5% CO_2_ for 2-3 hours in the dark. The absorbance at 450 nm was measured using a microplate reader. The mean optical density (OD, absorbance) of four wells in the indicated groups was used to calculate the relative OD value as follows: relative OD value = (A_treatment_ − A_blank_)/(A_control_ − A_blank_) × 100% (where *A* = absorbance).

### 2.4. TUNEL Assay

A TUNEL assay kit was used to measure apoptosis. Second passage astrocytic cells were seeded into a 24-well plate at a density of 0.5 × 10^5^ cells/well. When cultures reached approximately 70–80% confluency, complete medium was replaced with serum-free DMEM/F12 for 24 hours and cells were treated with different concentrations of SFN for 24 hours. The medium was then discarded and cells were rinsed with PBS. Cells were then fixed with 4% (w/v) paraformaldehyde for 30–60 minutes at room temperature. Following fixation, the paraformaldehyde solution was discarded and cells were rinsed with PBS. PBS containing 0.1% (w/v) Triton X-100 was then added, and the plate was placed on ice for 2 minutes. Cells were then rinsed with PBS twice, followed by addition of 50 *μ*l TUNEL reagent per well. Cells were incubated with TUNEL reagent at 37°C with 5% CO_2_ for 1 hour in the dark. Cells were then rinsed with PBS twice, followed by staining with DAPI. TUNEL and DAPI staining were visualized at wavelengths of 515–565 nm and 488 nm, respectively, using fluorescence microscopy. Immunofluorescence intensity was analyzed by ImageJ software.

### 2.5. Flow Cytometry

The FITC Annexin V Apoptosis Detection Kit I was used to measure cell apoptosis. Second passage astrocytic cells were seeded in 6-well plates at 5 × 10^5^ cells/well for each group for 24 hours. Cells were treated with different concentrations of SFN for 24 hours when fully attached. Both floating and adherent cells were collected and washed twice with cold PBS. Then, cells were resuspended in 500 *μ*l binding buffer, 5 *μ*l Annexin V-FITC, and 5 *μ*l propidium iodide (PI) and incubated in the dark at room temperature for 15 minutes. Cell apoptosis was detected by BD LSRFortessa X-20 and analyzed by FlowJo software.

### 2.6. Immunofluorescence

Immunofluorescence staining was carried out in order to study morphological changes of astrocytes. Second passage astrocyte cells were seeded into a 24-well plate at a density of 0.5 × 10^5^ cells/well. When astrocyte cultures reached 70–80% confluency, complete medium was replaced with serum-free DMEM/F12 for 24 hours, and cells were treated with different concentrations of SFN for 24 hours. Following SFN treatment, the medium was discarded and cells were rinsed with PBS. Cells were then fixed with 4% (w/v) paraformaldehyde for 15 minutes at room temperature. Following fixation, the paraformaldehyde solution was discarded and cells were rinsed with PBS for a total of three times. Cells were then incubated with a 0.1% (w/v) Triton X-100 solution containing 10% (v/v) goat serum for 30 minutes. Cells were then rinsed with PBS and incubated with GFAP and AQP4 primary antibodies (1 : 400) at 4°C overnight with gentle shaking. Next, cells were rinsed with PBS for a total of three times followed by incubation with AQP4 and GFAP secondary antibodies (1 : 300) at room temperature for 30 minutes in the dark. Cells were then rinsed with PBS for a total of three times and were then stained with DAPI. GFAP, AQP4, and DAPI staining were visualized using fluorescence microscopy at wavelengths of 617 nm, 519 nm, and 488 nm, respectively.

### 2.7. Western Blotting

Second passage astrocytic cells were seeded into a 6-well plate at a density of 0.3 × 10^6^ cells/well. Once astrocytic cultures reached 70–80% confluency, complete medium was replaced with serum-free DMEM/F12 for 24 hours and cells were treated with different concentrations of SFN for 24 hours. Following SFN treatment, the medium was discarded and cells were rinsed with PBS. A total of 150 *μ*l of RIPA lysis buffer was added to each well, and the plate was placed on ice for 20 min. Lysate was then centrifuged at 16000 ×g for 5 minutes. Following centrifugation, the protein concentrations were measured using a BCA protein assay kit. Samples were then subjected to SDS-PAGE electrophoresis (80 mV for 30 minutes, followed by 100 mV for 90 minutes). The gels of different target proteins were cut according to the size markers and then transferred to PVDF membrane at 250 mA for 2 hours. PVDF membranes were blocked with 5% bovine serum albumin (BSA) and incubated with specific primary antibodies overnight at 4°C, followed by incubation with horseradish peroxidase-conjugated secondary antibodies for 1 h at room temperature. Protein bands were visualized using a chemiluminescence detection kit. All bands were analyzed by ImageJ software.

### 2.8. Statistical Analysis

SPSS 20.0 software was used to carry out statistical analyses. Data are presented as the mean ± SD. All groups were compared by one-way analysis of variance (ANOVA) followed by Bonferroni with homogeneity of variance or Dunnett T3 with heterogeneity of variance. The difference was determined to be statistically significant with a *P* value < 0.05.

## 3. Results

### 3.1. Effects of SFN on Proliferation of Cultured Mouse Astrocytes

In order to screen for the appropriate SFN concentration and working time for our studies, a CKK-8 assay was utilized to analyze the effect of SFN on the proliferation of cultured mouse astrocytes. Astrocyte cultures were exposed to different SFN concentrations (0, 0.1, 0.25, 0.5, 2.5, 5, and 10 *μ*M) for 6, 12, and 24 hours.

The CKK-8 assay demonstrated significant differences among different working times and different concentrations of SFN (F_6 h_ = 19.914, *p*_6 h_ < 0.001; F_12 h_ = 207.290, *p*_12 h_ < 0.001; F_24 h_ = 188.821, *p*_24 h_ < 0.001) (Figure 2). Addition of SFN for 6 hours was found to result in an increase in relative OD value when added at concentrations of 0.1, 0.25, 0.5, 1, and 2.5 *μ*M, with no significant difference observed compared to the vehicle treatment group. However, the relative OD value was found to significantly increase when SFN was added to cultures for 12 hours at concentrations of 0.25, 0.5, 1, and 2.5 *μ*M SFN (*p*_0.25 *μ*M_ = 0.01，*p*_0.5*μ*M_ < 0.01, *p*_1 *μ*M_< 0.01, and *p*_2.5*μ*M_ < 0.01). In addition, the relative OD value was also found to significantly increase when treated with SFN for 24 hours at concentrations of 0.5 and 1 *μ*M (*p*_0.5*μ*M_ = 0.027, *p*_1 *μ*M_ = 0.018). Addition of 10 *μ*M SFN for 6, 12, and 24 hours was found to result in significantly decreased relative OD value compared to the vehicle treatment group (*p* < 0.01). According to the results described above, in our study, addition of 1 *μ*M SFN to astrocytes for 24 hours resulted in peak relative OD value. Therefore, we treated astrocytes with different concentrations of SFN for 24 hours in the following experiments.

### 3.2. Effects of SFN on Apoptosis of Cultured Mouse Astrocytes

TUNEL assay was utilized to investigate the effect of SFN treatment on apoptosis of cultured mouse astrocytes. When astrocytes were treated with 0, 1, and 5 *μ*M SFN for 24 hours, the TUNEL assay showed no significant difference of apoptotic cells in each group (Figure 3(a)). Flow cytometry also was used to detect cell apoptosis of astrocytes treated with 0, 1, and 5 *μ*M SFN for 24 hours. Results showed that there was no significant difference in normal cells (Q4), early apoptotic cells (Q3), and late apoptotic cells(Q2) in each group (Figure 3(b)∼3(e)). Using western blotting, we further tested for the activation of Caspase-3, a downstream apoptosis protease involved in the main signal transduction pathway of apoptosis. Activated Caspase-3 is known to be cleaved into different protein fragments, such as 17 KDa and 19 KDa molecular weight fragments that participate in apoptosis. Western blotting results demonstrated that cleaved Caspase-3 fragments were not formed, indicating that SFN does not induce apoptosis at a concentration of 5 *μ*M, in accordance with the results of TUNEL assay and flow cytometry (Figure 3(f)).

### 3.3. Effects of SFN on the Morphology of Cultured Mouse Astrocytes

Immunofluorescence was utilized to observe the morphological changes of cultured astrocytes (Figure 4(a)). Compared to the vehicle treatment group, cultured astrocytes treated with 1 *μ*M SFN were observed to proliferate vigorously and possess larger cell bodies as well as a greater number of astrocytic processes. Enhanced GFAP and AQP4 immunofluorescence staining was also observed with a 1 *μ*M SFN treatment (Figure 4(b)). When astrocytes were treated with 5 *μ*M SFN, shrinking cell body size was observed and showed decreased GFAP and AQP4 immunofluorescence staining relative to 1 *μ*M, however with no significant difference for 5 *μ*M compared to the vehicle group (Figures 4(a) and 4(b)).

### 3.4. Effect of SFN on AQP4 Expression and p38 MAPK Phosphorylation in Cultured Mouse Astrocytes

In addition to the immunofluorescence results demonstrating enhanced AQP4 immunofluorescence staining when cells were treated with a concentration of 1 *μ*M SFN, we further evaluated the effect of SFN on AQP4 expression in cultured mouse astrocytes using western blotting. Following treatment of astrocytes with different SFN concentrations for 24 hours, we observed significant differences in AQP4 expression among different treatment groups (*F* = 301.200, *p* < 0.001). Compared to the vehicle treatment group, we observed a significant enhancement of AQP4 expression in groups treated with 0.5 and 1 *μ*M SFN (*p*_0.5 *μ*M_ < 0.0001, *p*_1_*μ*_M_ < 0.0001) (Figures 5(a) and 5(b)). However, in the case of groups treated with 5 *μ*M SFN, we observed significantly lower AQP4 expression levels (*p* < 0.0001) (Figures 5(a) and 5(b)). In order to identify the potential mechanism of SFN in the upregulation of AQP4 expression in cultured mouse astrocytes, we treated astrocytes with different concentrations of SFN for 24 hours and examined p38 MAPK phosphorylation by western blotting (Figure 5). These results demonstrated a significant difference among different groups in the phosphorylation state of p38 MAPK (*F* = 460.000, *p* < 0.001). Western blotting demonstrated the detection of activated p38 MAPK upon treatment with 0.5, 1, and 2.5 *μ*M SFN (*p*_0.5 *μ*M_ < 0.05, *p*_1 *μ*M_ < 0.0001, and *p*_2.5 *μ*M_ < 0.0001) (Figures 5(a) and 5(c)). However, groups treated with 5 *μ*M SFN demonstrated a downregulation of p38 MAPK phosphorylation levels (*p* < 0.05) (Figures 5(a) and 5(c)). Therefore, we determined that SFN could function to upregulate p38 MAPK phosphorylation levels, a hypothesis consistent with changes in AQP4 expression levels. These results indicate that activation of p38 MAPK signaling pathway could likely play a role in the regulation of AQP4 expression.

### 3.5. SFN Upregulated AQP4 Expression in Cultured Mouse Astrocytes through p38 MAPK Pathway

SB203580 is a p38 MAPK pathway inhibitor, which inhibits the phosphorylation of activating transcription factor-2 (ATF-2), which is a downstream substrate of p-p38 [19]. In order to verify the role of the p38 MAPK signaling pathway in the regulation of astrocytic AQP4 expression, we pretreated astrocytes with the p38 MAPK pathway inhibitor, SB203580, for 2 hours prior to treatment with 1 *μ*M SFN (Figure 6). Compared to the vehicle treatment group, p38 MAPK phosphorylation levels in cells treated only with SB203580 demonstrated that SB203580 could function to significantly inhibit activation of p38 MAPK pathway (*p* = 0.021). Consistent with these previous results, a 1 *μ*M SFN treatment was found to significantly upregulate astrocytic AQP4 expression as well as p38 MAPK phosphorylation levels compared to the vehicle treatment group (*p* < 0.01). When cells were pretreated with SB203580 for 2 hours prior to treatment with 1 *μ*M SFN, the upregulation of astrocytic AQP4 expression and the phosphorylation levels of p38 MAPK were found to be alleviated compared to the group treated with only 1 *μ*M SFN. Therefore, we demonstrate that SB203580 functions to reverse the upregulation effect of SFN on astrocytic AQP4 expression. This indicates that SFN could function to upregulate astrocytic AQP4 expression through p38 MAPK signaling pathway.

## 4. Discussion

This study aimed to evaluate the effect of SFN, along with its underlying mechanism, on the regulation of AQP4 expression in cultured mouse astrocytes. Our results demonstrated that SFN caused hormesis effect on cultured mouse astrocytes. We demonstrated that SFN treatment resulted in an upregulation of astrocytic AQP4 expression by acting through p38 MAPK pathway. These results suggest that SFN could be utilized as a potential drug to accelerate protein clearance via AQP4 mediated pathways in parenchyma. Such a drug might be used for the prevention and treatment of neurodegenerative diseases including AD in the future.

SFN has been demonstrated to have extensive pharmacological effects, including antitumor, antioxidant, and neurological protection properties [20]. Prior studies regarding SFN demonstrated that its pharmacological effects showed an obvious dose-response relationship. At low doses, SFN was shown to promote cell grow, proliferation, and differentiation. At high doses, SFN was shown to be toxic to cells, resulting in cell cycle arrest, apoptosis, and senescence [21–23]. Thus, SFN exhibits different biological effects depending on the concentration cells are treated with. This is referred to as the hormesis effect [21]. In our study, we demonstrated that SFN functioned to promote proliferation of astrocytes when treated at low doses (such as 1 *μ*M and 2.5 *μ*M), while treatments at high doses (such as 5 *μ*M and 10 *μ*M) resulted in suppressed proliferation. Therefore, we found that SFN displays significant hormesis effect in our studies as well. Surprisingly, in our study, we did not find that SFN induced apoptosis in treated astrocytes, which was demonstrated in treated astrocytoma, multiple myeloma cells, prostate cancer cells, and so on in previous studies [24–26]. These disparate results could be attributed to the cells that were investigated, as well as the exerting time and/or concentration of SFN used.

Astrocytes are the primary glial cells in the mammalian brain and play a critical role in the maintenance of homeostasis in the central nervous system [27]. Astrocytes function to maintain the balance of water, electrolytes, and neurotransmitters, regulate signal transduction of neurons, and secrete nerve growth factors, including brain-derived neural factor and glial-derived neural factor [11]. In addition to maintaining a stable internal environment to protect the brain, astrocytes can be activated to protect the brain from harmful factors as well. Activated astrocytes exhibit a larger cell body with a greater number of processes and increased GFAP expression, which is referred to as astrogliosis [28]. Astrogliosis can function to provide nutritional support and neuroprotection, isolate damage from the other parenchyma, reconstruct the BBB function, and regenerate damaged areas [29]. Studies have shown that astrogliosis plays a role in neurodegenerative diseases, such as AD [28] and amyotrophic lateral sclerosis (ALS) [30–32]. Astrogliosis exhibits a neuroprotection effect in the early stage of diseases. However, as astrogliosis progresses, it causes harmful effects on cell metabolism, neurovascular units, neuroglial network, and synapse dysfunction, resulting in progressive cognitive decline [29]. In our study, we demonstrate that low dose of 1 *μ*M SFN could function to activate astrocytes. These astrocytes exhibited a larger cell body, a greater number of processes, and enhanced GFAP fluorescence staining. Meanwhile, there was a tendency of decreased GFAP immunofluorescence staining along with shrinking cell body size when astrocytes were treated with a high dose of 5 *μ*M SFN, indicating that SFN may exert some toxic effects although SFN did not induce apoptosis in treated astrocytes in our study, and further works are needed to investigate the underlying mechanisms. In AD, it is thought that, in the early stages, activated astrocytes are beneficial to A*β* degradation and clearance, thereby functioning to prevent the accumulation of A*β* in parenchyma.

In addition to the activation of astrocytes, treatment with low doses of SFN was also found to enhance AQP4 immunofluorescence staining and expression levels. As the most highly expressed aquaporin in the mammalian brain, AQP4 primarily distributes on the endfeet of astrocytes [11]. The primary function of AQP4 is to facilitate water movement across the plasma membrane driven by osmotic gradients and hydrostatic gradient, thus maintaining the water balance of cells [33]. AQP4 is known to play a critical role in the maintenance of astrocytic functions and is associated with astrocytic polarity [11]. Studies have shown that astrocytes are limited in proliferation, activation, and forming glial scar in *AQP4*-knockout mouse in cranial and spinal injury [34]. This indicates that AQP4 plays a role in the regulation of astrocyte activation. Therefore, increased AQP4 expression levels could function as a marker for astrocyte activation. AQP4 plays a key role in CNS entities such as encephaledema, brain tumor, epilepsy, and neuromyelitis optica [12]. Besides, AQP4 is thought to play a role in neurodegenerative diseases, including AD, PD, and ALS. For example, in AD, AQP4 is known to play a role in A*β* clearance, synapse function, transportation of potassium and sodium, and inflammation reactions [5, 13, 35]. In the case of ALS, AQP4 dysfunction has been linked to a disturbance in water and potassium balance, leading to BBB dysfunction, internal environment disorder, and neuron dysfunction and death [36]. Notably, accumulating studies have demonstrated that AQP4 plays an important role in glymphatic system, whose waste clearance function is based on the AQP4-dependent trans-astrocytic ISF bulk ﬂow [7]. Study has shown that the interstitial clearance rate of the glymphatic pathway is reduced by approximately 70%, resulting in a 55% reduction in A*β* clearance in AQP4-null mice [7]. Therefore, considering the critical role of AQP4 in the clearance systems in brain, an understanding of its regulation mechanisms is of critical importance in the therapy field of the protein clearance dysfunction related neurodegenerative disease.

Numerous factors have been shown to regulate AQP4 expression levels, including transcriptional, translational, and posttranscriptional modification processes [37]. Previous studies have shown that SFN could function to upregulate AQP4 expression levels in TBI animal models, resulting in relieving cerebral edema [18]. However, the underlying mechanism surrounding this process is unclear. Mitogen-activated protein kinases (MAPKs) are a family of serine/threonine protein kinases, which mainly include extracellular signal-regulated kinase (ERK), c-Jun N-terminal kinase (JNK), and p38 MAPK, mediating various cellular responses to external stressors, such as stress responses, apoptosis, and immune defense [38, 39]. MAPKs also participate in the development of reactive gliosis [40]. The p38 MAPK pathway is an important part of MAPKs signaling transduction pathways and plays roles in regulating the inflammatory response, tau protein phosphorylation, and synaptic plasticity in glial cells [41]. Previous studies have shown that p38 MAPK is involved in regulating AQP4 in different CNS disease models, such as ischemic [42], intracerebral hemorrhage (ICH) [43], traumatic brain injury [44], epilepsy [45], glioma [46], and carbon monoxide (CO) poisoning [47]. Although certain studies have all demonstrated that upregulation of AQP4 expression is via p38 MAPK pathway [43, 45, 47], the biological effects of upregulated AQP4 are different due to different CNS disease models. For example, study showed that the overexpressions of AQP4 were involved in the development of CO poisoning-induced cerebral oedema through p38 MAPK signaling in rat astrocytes [47], while another study showed that Erythropoietin (EPO) protects BBB from disruption after ICH is associated with increased levels of AQP4 through activation of p38 MAPK pathways after binding to EPOR [43]. Our research has shown that, at a proper concentration (e.g., 1 *μ*M), SFN can function to significantly upregulate AQP4 expression and p38 MAPK phosphorylation levels. In addition, we show that the p38 MAPK pathway inhibitor (SB203580) could reverse these effects, demonstrating that SFN upregulated AQP4 expression via p38 MAPK pathway. However, the underlying mechanism on how p38 MAPK pathway is involved in the regulation of AQP4 expression is still unclear. Study has shown that phosphorylated p38 MAPK activates I*κ*B kinase and leads to activation of NF-*κ*B, a critical transcription factor involved in the transcription of many genes associated with inflammation [48]. AQP4 expression would be reduced by inhibiting the activation of NF-*κ*B [49], which indicates the important role of NF-*κ*B in regulating AQP4 expression and may be associated with production of proinflammatory cytokines. Further studies are required to gain deeper understanding of the underlying mechanism between p38 MAPK pathway and the regulation of AQP4 expression.

Clearance of misfolding and/or aggregated protein in brain at the early stage of diseases is one of the therapy strategies for neurodegenerative diseases. In AD patients, A*β* deposition is thought to be followed by hyperphosphorylation and aggregation of tau protein and neurodegeneration some 10 to 20 years later and closer to clinical disease onset [50, 51]. The recent version of the A*β* cascade hypothesis argued that imbalance between the production and the clearance of A*β* results in increased small soluble A*β*, leading to synapse failure and cognitive decline in AD patients [52, 53]. Thus, novel targets enhancing A*β* clearance may be future strategies for AD treatment. Preclinical neuroprotective evidence and plausible mechanisms of SFN in AD have been widely investigated in animal and cell models, suggesting that sulforaphane has a multiple neuroprotective effect on AD pathophysiology regarding amyloid-*β*, tau, inﬂammation, oxidative stress, and memory impairment [52, 53]. However, there are few studies focusing on the effect of SFN in the clearance system of brain. Taken together, the above results in our study shed new lights on novel targets such as the fact that SFN could be used to upregulate AQP4 expression, which could result in enhanced soluble protein clearance through AQP4-mediated glymphatic pathways and be of great importance in the treatment of protein misfolding diseases, such as the early stage of AD.

However, we note that there exist some limitations to our study. Firstly, our study utilizes cultured astrocytes as the experimental subject. However, we recognize that cultured astrocytes differ from astrocytes *in vivo* [56]. Noticeably, AQP4 is mainly distributed in the endfeet of astrocytes in parenchyma *in vivo*, while AQP4 is distributed uniformly in cultured astrocytes [57]. In order to mimic the internal environment, a coculture model of astrocytes together with endothelial cells, or brain slice culture, or an animal model could be used to further validate the findings from this study. In addition, we suggest that SNF functions to upregulate AQP4 expression in astrocytes via p38 MAPK pathway. This merely provides the possibility that SFN could affect the clearance of the A*β*, tau, and other soluble proteins. Further animal studies are needed to validate these findings as well [54, 55].

## 5. Conclusion

Our findings demonstrate that SFN exerts hormesis effect on cultured mouse astrocytes, and SFN can function to upregulate astrocytic AQP4 expression via p38 MAPK pathway. Further studies are needed in order to verify these findings *in vivo* and to evaluate the potential role of SFN in the clearance of soluble proteins in brain.

## Figures and Tables

**Figure 1:** Identification of cultured mouse astrocytes by immunofluorescence. Immunofluorescence was utilized to identify the second passage astrocytes with the specific marker of the astrocytes, glial fibrillary acidic protein (GFAP). It showed that the cultured astrocytes are GFAP (+) cells with different sizes and shapes. Statistically, the purity of the cultured astrocytes was more than 99%, a level suitable for experiments.

**Figure 2:** Effect of SFN on the proliferation of cultured mouse astrocytes by CCK-8. Astrocytes were treated with different concentrations of SFN for 6, 12, and 24 hours. The CKK-8 assay demonstrated significant differences among different working times with different SFN concentrations. When 1 *μ*M SFN was added to astrocyte for 24 hours, the relative OD value of astrocytes was found to reach the peak value in our study. Compared to the vehicle treatment group, ^*∗*^*p* < 0.05,^#^*p* < 0.01.

**Figure 3:** Effect of SFN on apoptosis of cultured mouse astrocytes. (a) TUNEL assay showed no significant difference in cell apoptosis among astrocytes treated with 0, 1, and 5 *μ*M SFN for 24 hours. (b–e) Flow cytometry showed no significant difference in normal cells (Q4), early apoptotic cells (Q3), and late apoptotic cells (Q2) among astrocytes treated with 0, 1, and 5 *μ*M SFN for 24 hours. Q1:(Annexin V-FITC)-/PI+; Q2: (Annexin V + FITC)+/PI+; Q3: (Annexin V-FITC)+/PI-; Q4: (Annexin V-FITC)-/PI-. (f) Western blotting testing the activation of Caspase-3. The result showed that no cleaved Caspase-3 fragments (17 KDa and 19 KDa molecular weight) were detected among astrocytes treated with 0, 1, and 5 *μ*M SFN for 24 hours.

**Figure 4:** Effect of SFN on morphological changes in cultured mouse astrocytes. (a) Immunofluorescence showed morphological changes of cultured astrocytes treated with 0, 1, and 5 *μ*M SFN. The cultured astrocytes were vigorously proliferated with larger cell bodies and a greater number of astrocytic processes treated with 1 *μ*M SFN and showed a shrinking cell body size when treated with 5 *μ*M SFN. (b, c) Quantitative analysis for GFAP (b) and AQP4 (c) staining of astrocytes. Results showed enhanced GFAP and AQP4 immunofluorescence staining when treated with 1 *μ*M SFN. When treated with 5 *μ*M SFN, they showed decreased GFAP and AQP4 immunofluorescence staining, however with no significant difference compared to the vehicle group. ^*∗*^*p* < 0.05,^∗∗^*p* < 0.01.

**Figure 5:** Effect of SFN on AQP4 expression and phosphorylation of p38 MAPK of cultured mouse astrocytes by WB. (a) Effect of SFN on AQP4 expression and phosphorylation of p38 MAPK of cultured mouse astrocytes by WB. (b, c) Quantitative analysis for AQP4 expression (b) and phosphorylation of p38 MAPK (c). Western blotting showed significant increase in AQP4 expression in groups treated with 0.5 and 1 *μ*M SFN for 24 hours compared to the vehicle treatment group, while the groups treated with 5 *μ*M SFN showed significantly decreased AQP4 expression. Meanwhile, western blotting showed significant increase in phosphorylation of p38 MAPK in groups treated with 0.5, 1, and 2.5 *μ*M SFN for 24 hours compared to the vehicle treatment group, while the groups treated with 5 *μ*M SFN showed significantly decreased phosphorylation of p38 MAPK. Compared to the control group, ^*∗*^*p* < 0.05,^∗∗∗∗^*p* < 0.0001.

**Figure 6:** The p38 MAPK inhibitor (SB203580) attenuated the upregulated expression of AQP4 and the phosphorylation of p38 MAPK pathway of cultured mouse astrocytes treated with 1 *μ*M SFN. (a) Effect of SB203580 on the expression of AQP4 and the phosphorylation of p38 MAPK. (b, c) Quantitative analysis for AQP4 expression (b) and phosphorylation of p38 MAPK (c). Astrocytes were pretreated with p38 MAPK pathway inhibitor, SB203580 (10 *μ*M), for 2 hours prior to treatment with 1 *μ*M SFN. The level of p38 MAPK phosphorylation in the group treated with SB203580 decreased. Astrocytic AQP4 expression and p38 MAPK phosphorylation level were found to be significantly upregulated in the 1 *μ*M SFN treatment group compared to the vehicle treatment group. The upregulated expression of astrocytic AQP4 and phosphorylation level of p38 MAPK were found to be attenuated compared to the group treated with 1 *μ*M SFN when SB203580 was pretreated. ^*∗*^*p* < 0.05,^∗∗∗∗^*p* < 0.0001.

## Data Availability

All the data are shared in the main manuscript.
